This article has been retracted.

# Design of Financial Management Model Using the Forward Neural Network Based on Particle Swarm Optimization Algorithm

**DOI:** 10.1155/2022/7536492

**Published:** 2022-01-30

**Authors:** Yilin Pan

**Affiliations:** Zhejiang University of Finance & Economics Dongfang College, Haining, Zhejiang 310012, China

## Abstract

The financial crisis of listed companies will bring huge losses to investors, so it is very important to establish a financial early warning model for investors and other stakeholders. The forward neural network model of particle swarm optimization is used to model and analyze the financial early warning of listed companies. In terms of data selection, earnings management indicators are substituted into the model for the common phenomenon of earnings management in listed companies. The results show that the accuracy of the model considering earnings management factors is improved from 65% to 70%. In the process of modeling, this paper uses the logistic regression model to further modify the model. The empirical results show that the accuracy of the model can be improved from 70% to 75%. When using the forward neural network model based on particle swarm optimization to make an empirical analysis of financial early warning of listed companies, adding quantitative indicators of earnings management can improve the accuracy of the model. In the demonstration, the correction of logistic regression model can also improve the accuracy of the particle swarm neural network financial early warning model. This greatly reduces the risk that companies with poor financial conditions will face bankruptcy and liquidation.

## 1. Introduction

In recent years, with the rapid development of the financial market, the securities market has become the central hub of financing and investment, and listed companies, as the cornerstone of the whole capital market, play an increasingly important role [1]. However, listed companies may also have certain business risks. From the external environment, changes in the macroeconomic environment and industry will bring many risk factors to the company [2]. From the perspective of internal environment, problems such as management turbulence may also bring certain risks to the company's internal governance [3]. To some extent, the risk factors of listed companies can be experienced through financial data. Investors will also determine their own investment strategy according to the financial data of listed companies, and the regulatory authorities will monitor the financial data of listed companies [4]. The company law stipulates that if a listed company has suffered losses for three consecutive years, the regulatory authority will suspend the company's stock sales and limit a period of time to rectify the company. If the rectification fails to meet the requirements within this period, the company's stock sales will be terminated [5]. The CSRC decided to label companies with abnormal financial conditions with “ST,” and the policy intervention accelerated the survival of the fittest in the securities market. Financial crisis can be predicted in advance [6]. By establishing an effective and accurate financial early warning mechanism, listed companies can predict the real financial situation in advance and then correct the company's strategy in time through internal rectification, so as to avoid further deterioration [7]. Investors can also select stocks and bonds worthy of investment according to the financial early warning model [8]. Therefore, this paper will try to establish an effective financial early warning model.

The innovation of this paper is to use the forward neural network model based on particle swarm optimization to make an empirical analysis of financial early warning of listed companies. The forward neural network model of particle swarm optimization is used to model and analyze the financial early warning of listed companies. In terms of data selection, earnings management indicators are substituted into the model for the common phenomenon of earnings management in listed companies. In the demonstration, the modification of logistic regression model can also improve the accuracy of the particle swarm optimization neural network financial early warning model. This greatly reduces the risk of bankruptcy and liquidation of companies with poor financial conditions.

This paper is divided into five chapters. Chapter 1: the research background of financial early warning model is introduced. Chapter 2: the research status of the existing financial early warning model is discussed. Chapter 3: the theoretical part of forward neural network model optimized by particle swarm optimization algorithm is described. Chapter 4: empirical analysis in MATLAB software is done, quantitative factors of earnings management is added, and the logical regression model to modify the forward neural network model based on particle swarm optimization is implemented. Chapter 5: this paper is concluded.

## 2. Related Work

In the research of financial forecasting modeling, the corresponding financial forecasting is mainly through the construction of neural network models. Models such as SVM model and decision tree have been gradually used [9]. The first stage of financial forecasting model proposed by scholars is from 1930s to 1980s. The research at this stage is limited by the lack of computing power. They mainly use a single index to model the enterprise and establish a prediction model based on a small number of samples. In 1932, Fitzpatrick conducted corresponding research on 19 companies through a single variable for the first time. By comparing the different financial ratios of successful companies and failed companies, he tried to find out the important factors determining the success or failure of companies. Finally, he thought that the shareholder's equity liability ratio and the return on net assets were two important indicators to distinguish the financial risks of enterprises [10]. The second stage was from 1980s to the beginning of the 21st century. In this stage, with the development of machine models and the improvement of computer hardware performance, new technical methods such as logistic regression were applied to the study of financial models, and the indicators used in financial modeling were also changed, and the number of research samples has increased to hundreds or even thousands [11–14]. The third stage is from the beginning of the 21st century to the present. With the vigorous development of various neural network models, the field of financial analysis has gradually begun to try to combine neural network models with financial analysis. More complex models have been constructed, and the accuracy of the models has been further promoted. In 2000, Charalambous et al. built a financial crisis warning model based on a sample of American companies from 1983 to 1994 on the basis of option pricing theory and explained corporate bankruptcy. The results of the model indicated that the main option incentive variables (such as corporate performance volatility) played an important role in predicting defaults in the first, two, and three years of bankruptcy [15]. Ptak-Chmielewska built a bankruptcy prediction model based on the SVM algorithm. By comparing three typical corporate distress models with this model, they concluded that traditional neural network algorithms can effectively predict corporate distress from the perspective of financial statements [16]. Zhou et al. discussed the effectiveness and limitations of SVM when applied to the bankruptcy prediction problem, and the experimental results showed that the SVM method of their classifier performed better than the BPN neural network model on corporate bankruptcy problems, and with the reduction of the training set size, the accuracy and generalization degree of the SVM algorithm are higher than those of the BPN algorithm [17]. Zelenkov et al. proposed the two-step classification method (TSCM) and built a related enterprise crisis warning model. They tested some companies using financial ratio indicators, and a lot of indicator training models including economic indicators and microeconomic indicators have obtained the ideal accuracy rate [18]. In the research on financial indicators to construct forecasting models, the related research started early and mainly experienced three stages, from single-variable modeling to multivariable modeling, and then to the use of machine learning to build financial forecasting models. With the progress of academic level and the development of scientific and technological strength, various traditional machine learning models and new neural network models have been widely used in financial forecasting models [19–23].

## 3. Forward Neural Network Model Based on Particle Swarm Optimization

Let the position vector *X*_*i*_ and velocity vector *V*_*i*_ of the *i* particle in the particle swarm optimization algorithm represent *X*_*i*_=(*x*_*i*1_, *x*_*i*2_, *x*_*i*3_,…, *x*_id_) and *V*_*i*_=(*v*_*i*1_, *v*_*i*2_, *v*_*i*3_,…, *v*_id_), respectively, the best position vector *P*_*i*_=(*p*_*i*1_, *p*_*i*2_, *p*_*i*3_,…, *p*_*i*  *d*_) of the *i* particle, and the best position vector *P*_*g*_=(*p*_*g*1_, *p*_*g*2_, *p*_*g*3_,…, *p*_*g*  *d*_) of the population. The position component of each particle represents the weight and threshold of the forward neural network. Note that the number of nodes in the input layer, middle layer, and output layer of the forward neural network model are *n*_*i*_, *n*_*h*_, and *n*_0_, respectively. The *i* particle determines the network according to the following:

(1) $$\begin{array}{c} X_{i}=\left(x_{i1},x_{i2},x_{i3},\ldots ,x_{\text{id}}\right)=\left(\omega_{11},\omega_{12},\ldots ,\omega_{n_{0}n_{h}},\;\mu_{11},\mu_{12},\ldots ,\mu_{n_{h}n_{i}},\;\sigma_{1},\sigma_{2},\ldots ,\sigma_{n_{0}},{\hat{\sigma }}_{1},{\hat{\sigma }}_{2},\ldots ,{\hat{\sigma }}_{n_{h}}\right). \end{array}$$

*ω*_12_ and *μ*_12_ are the weights from the middle layer to the output layer and from the input layer to the middle layer node, respectively, and *σ*_1_ and ${\hat{\sigma }}_{1}$ represent the thresholds of the output layer node and the middle layer node, respectively.

Make *γ*_1_=*n*_0_*n*_*h*_,  *γ*_2_=*γ*_1_+*n*_*h*_*n*_*i*_,  *γ*_3_=*γ*_2_+*n*_0_,  *γ*_4_=*γ*_3_+*n*_*h*_. Then, the update formula of the position of the second particle is (2) and (3):

(2) $$\begin{array}{c} v_{im}\left(s+1\right)=\eta *v_{im}\left(s\right)+c_{1}r_{1}\left(p_{im}-x_{im}\left(s\right)\right)+c_{2}r_{2}\left(p_{gm}-x_{im}\left(s\right)\right), \end{array}$$

(3) $$\begin{array}{c} x_{im}\left(s+1\right)=\left\{\begin{array}{c} x_{im}\left(s\right)+v_{im}\left(s+1\right)+\alpha \delta_{k}H_{j_{1}},\;m\in \left(0,\gamma_{1}\right],\\ x_{im}\left(s\right)+v_{im}\left(s+1\right)+\alpha \sigma_{j_{2}}I_{h},\;m\in \left(\gamma_{1},\gamma_{2}\right],\\ x_{im}\left(s\right)+v_{im}\left(s+1\right)+\beta \delta_{k_{1}},\;m\in \left(\gamma_{2},\gamma_{3}\right],\\ x_{im}\left(s\right)+v_{im}\left(s+1\right)+\beta \delta_{j_{3}},\;m\in \left(\gamma_{3},\gamma_{4}\right]. \end{array}\right. \end{array}$$

There is

(4) $$\begin{array}{c} m=1,2,\ldots ,d,k=\left[\frac{m}{n_{h}}\right],\\ j_{1}=m-\left(k-1\right)*n_{k},\\ j_{2}=\left[\frac{m-l_{1}}{n_{i}}\right],\\ h=m-\gamma_{1}-\left(j_{2}-1\right)*n_{i},\\ k_{1}=m-\gamma_{2},j_{3}=m-\gamma_{3}. \end{array}$$

The specific steps are divided into three stages. First, initialize the model:

(l) Initialize the parameters of the forward neural network model, including the number of nodes in the input layer, middle layer, and output layer, learning rate *α*, *β*, and so on
(2) Initialize particle swarm parameters, including particle swarm number, accuracy requirements, constant coefficient, inertia weight, and iteration times

Second, the model is updated iteratively: the above formula is used to update the speed and position of each particle. If the speed is greater than the maximum speed, the latest speed is assigned to the maximum speed. On the contrary, the maximum speed remains unchanged. Calculate the fitness of each particle as shown in the following:

(5) $$\begin{array}{c} f_{i}=\frac{1}{n}\sum_{q=1}^{n}{\left(O_{iq}-T_{iq}\right)}^{2}, \end{array}$$

where *n* is the number of training samples and *O*_*iq*_ − *T*_*iq*_ is the difference between the output value of the forward neural network and the actual value of the weight and threshold of the training sample *q* under the position vector of the *i* particle.

Each particle is calculated, and the minimum value of all individual extreme values is the global extreme value [24–28]. When the global extreme value is less than the accuracy requirements of the forward neural network or reaches the maximum number of iterations, the cycle is ended, otherwise the iteration is continued. The global extreme value is obtained, and the weight and threshold of the forward neural network are determined. Therefore, although the structure diagram of the forward neural network based on PSO algorithm is similar to that of the forward neural network, the function will be improved. Based on the PSO algorithm, the structure diagram of the forward neural network is shown in Figure 1.

## 4. Empirical Analysis

### 4.1. Data Preprocessing

The interval span of each indicator data in the data set is very different. The interval span of each index is shown in Figure 2.

In order to eliminate the interference caused by the large interval between indicators on subsequent experiments, the following methods are adopted for correction: suppose the *i* index *m*_*i*_=max{max_*i*_, −1*∗*min_*i*_}. Let the value of *j* of each element in *i*, newvalue_*j*_=value_*j*_/*m*_*i*_*∗*10 where value_*j*_ is the original value of *j* of *i* index. Through the above processing, the span of each index interval in the data set is controlled at [−10, 10], so that the model parameters are greatly disturbed by different interval values during subsequent model training, and the performance of the model is improved.

In addition, the market law determines that the number of high-quality enterprises that can quickly reverse their performance in the context of economic crisis is significantly less than that of other enterprises, so there is an inevitable problem of data imbalance in the sample, that is, the data sample marked “1” is significantly less than the data sample marked “0.” In order to avoid the problems of validity and practicability of prediction results caused by data imbalance, SMOTE (synthetic minority oversampling technology) algorithm is adopted to process the data set. The SMOTE algorithm is to extract *k* random samples from the nearest *n* samples and obtain new samples through interpolation. The SMOTE core formula is as follows:

(6) $$\begin{array}{c} Y_{\text{new}}=Y_{0}+\text{rand}\left(0,1\right)*\left(Y_{i}-Y_{0}\right),\text{ i}\in \left[1\text{,k}\right]. \end{array}$$

After data preprocessing, the total number of high-quality enterprises and other enterprises is close to 1 : 1, and the resulting data set is shown in Figure 3.

In addition, considering the performance of the model in terms of precision and recall, F1-score is used to investigate the model performance when center = 50, center = 200, and center = 500, respectively. From the experimental results, the model F1-score with beta coefficient less than 1 is significantly better than F1-score with beta coefficient greater than 1, and the optimal value of F1-score appears when beta = 0.1. Therefore, beta = 0.1 is used to test the center coefficient of the model. The specific experimental results of beta under different center values are shown in Figure 4.

### 4.2. Preliminary Adjustment Process of Forward Neural Network Based on Particle Swarm Optimization

Based on the good global optimization performance of PSO algorithm, this paper uses the PSO algorithm to optimize the neural network model. The performance of particle swarm optimization algorithm is improved by finding a better clustering radius and clustering center. In order to carry out subsequent experiments based on effective clustering radius, this section first calculates the Euclidean distance between sample points and counts the number of distances between samples in different intervals. According to the calculation results, the farthest distance between samples is 13.5. Therefore, we can divide the Euclidean distance between samples into 300 intervals in the unit of 0.1 and then calculate the sample quantity proportion and cumulative proportion in each interval, respectively. The results are shown in Figure 5. According to the statistical results, the distance relationship pairs in the [0.0, 3.0] interval account for 70.84% of the total relationship pairs. This interval covers more than 2/3 of the distance relationship pairs, which can basically meet the effectiveness requirements of subsequent clustering experiments. Therefore, specifying the interval [0.0, 3.0] as the clustering radius can effectively meet the subsequent experiments.

In the specific experiment, the clustering radius *R* is given, and an empty tabu table a is created. Traverse the experimental samples. When encountering the point a that is not included in the tabu table, add a to the tabu table, and create a new class to include a and define it as the center of the class. Then, traverse all points that are not included in the tabu table. If a point whose distance from the cluster center does not exceed R is encountered, add the point to the tabu table and include it in this class, and then update the cluster center according to all points in the class.

The above clustering experiments are carried out on the training set, and DI and DBI are used as evaluation indexes. In order to further improve the performance of the model, improve the global optimization ability of the algorithm, and avoid the algorithm falling into local optimization, a two-dimensional probability transfer matrix C1 is introduced for subsequent experiments. Assuming that the sample data have *N* entries and the clustering radius is R, the probability transfer matrix C1 is a matrix of N*∗*N, in which the a column in the a row of the probability matrix C1 (0 < a < N+1, 0 < b < N+1) represents the distance between the a sample point and the b sample point. The probability transfer matrix C1 is a Boolean two-dimensional matrix. If the distance between two sample points is less than the clustering radius R, the point in the probability matrix is marked as 1, otherwise it is marked as 0.

The probability transfer matrix C2 is established according to the probability transfer matrix C1, in which each point of the two-dimensional probability transfer matrix C2 of N*∗*N is calculated according to the point value in C1 divided by the column value, so it can be deduced that the sum of each column of C2 is 1. Compared with the first clustering algorithm, the improved clustering algorithm does not necessarily select the point when the algorithm traverses to a qualified point but selects the point with the corresponding probability in the probability transfer matrix C2. This processing method makes the program jump out of the local optimal solution to a certain extent and get the global optimal solution more easily. In the above experiments, the convergence speed of the ant colony algorithm is too slow. Combined with the sample data of the training set, due to the large amount of sample data, the probability of selecting the points that meet the clustering conditions in the probability transfer matrix C2 is very small, which leads to the slow convergence of the ant colony algorithm. On the other hand, the algorithm uses separate calculation when selecting each point. So it is almost difficult to select a point for clustering in the initial stage, which also leads to too slow convergence speed. In combination with the above characteristics, the probability transfer formula is modified as follows:

(7) $$\begin{array}{c} \tau_{ij}\left(t\right)=c*\frac{p_{ij}\left(t\right)}{\max_{1\leq j\leq k}p_{ij}\left(t\right)}. \end{array}$$

Here, 1 < c < 0. At the same time, in order to maintain the characteristics of probability transfer, the probability transfer matrix C1 is modified from Boolean matrix to floating-point matrix, and the corresponding probability of two sample points whose distance is less than the clustering radius R is also modified to c. In addition, in order to strengthen the characteristics of global optimization and positive feedback of the algorithm, the volatilization coefficient *ρ* and positive feedback mechanism are specified—when each cycle ends, increase the weight of the selected paths in this cycle, and make all paths volatilize according to the volatilization proportion coefficient *ρ* after all modifications. In addition, in order to avoid the situation that a point in the probability transition matrix is extremely difficult to be selected due to its low value, the lowest transition probability p1 is set to improve the probability that the point is selected, which also helps the algorithm jump out of the local optimal situation. In the specific experiment, there are three parameters: transfer probability c, volatilization coefficient *ρ*, and transfer probability p1 at the same time. At the same time, the ergodic test of these three parameters takes a long time, and at the same time, these three parameters have certain regularity when they change in a certain interval. Therefore, it is advisable to roughly calculate the transfer probability c, the volatilization coefficient *ρ*, and the transfer probability p1 are in the appropriate value range, and then a more accurate comparison is made to determine the parameter values of the transfer probability c, the volatilization coefficient *ρ*, and the transfer probability p1.  Figure 6 is the parameter curve of transition probability.

From the experimental results, the performances of model DBI and DI under different transition probability parameters c are different to a certain extent, but there is little difference on the whole. The difference between each group is more likely to be caused by the value of clustering radius R. If the DBI value and DI value under each transition probability parameter c are comprehensively evaluated without clustering radius CC, the performance of curves in each group will approach. However, different values of transition probability parameters have a significant impact on the convergence speed of the model, and the comprehensive performance of the model is better in the [0.8, 0.9] interval. From the experimental results, in the forward neural network based on particle swarm optimization, the value of TP type is 4217, the value of FN type is 1782, the value of FP type is 3608, and the value of TN type is 3947.

### 4.3. Practical Application of Forward Neural Network Model Based on PSO in Financial Management Model

In terms of sample selection, there are about 3000 listed companies, of which about 70 are ST stocks. This paper selects 100 listed company stocks (including 50 ST stocks and 50 non ST stocks) as training samples and 20 listed company stocks (including 10 ST stocks and 10 non ST stocks) as test samples to test the accuracy of the model. However, since the 2017 annual report is not fully disclosed, ST stocks and non-ST stocks in the market are the financial data as of 2016. In order to make the model more predictive, this paper selects these training samples and test sample companies' index data three years ago, that is, 2013. This paper selects 12 financial indicators from five aspects: solvency, asset operation ability, profitability, development ability, and cash flow. Earnings management indicators are added to offset the impact of earnings manipulation on the accuracy of the model. This paper uses the logistic regression model to modify the particle swarm neural network model, so as to improve the accuracy of the model. To some extent, the company's financial indicators can reflect the problems existing in the company's operation. As mentioned above, this paper selects financial indicators from two aspects: solvency and asset operation ability.

Earnings management can be divided into disclosure management and real earnings management. Disclosure management refers to earnings management realized by accounting means. For example, the company changed the depreciation method of fixed assets from accelerated depreciation method to average life method, so as to increase the profit of this year. Real earnings management refers to some real transactions deliberately carried out by the company's management in order to increase or reduce profits but harmful to the company's long-term development, such as significantly reducing R & D expenses and marketing expenses to increase account profits. The management of listed companies often uses these two methods to manipulate earnings in order to achieve certain purposes (such as affecting the company's stock price, improving their own remuneration, reducing the possibility of violating the loan treaty, or avoiding the intervention of regulatory authorities).

Disclosure management is a common method of earnings management of listed companies because it complies with accounting standards and will not have regulatory risks. The real earnings management is relatively hidden, but usually when the management arranges some transactions that do not comply with the company's long-term development strategy, it may meet the resistance of the company's board of directors. Moreover, the reduction in R & D expenses and marketing expenses will be reflected in the statements, which will arouse the suspicion of investors. Therefore, the real earnings management will be less than the disclosure management in terms of amount and frequency.

This paper considers the impact of two types of earnings management on the financial early warning model. The goal of earnings management is generally to increase or reduce the net profit of the income statement, but the cash flow of operating activities in the cash flow statement is composed of real transactions with poor controllability, which can objectively reflect the real operating conditions of the company to a certain extent. Therefore, the difference between net profit and cash flow from operating activities represents the degree of earnings manipulation of the company, which is standardized by dividing by total assets, so it is comparable.

The *p* value refers to the output result of the logistic regression model. A logistic regression model is established for the samples and financial indicators mentioned above to obtain the possibility of financial crisis of the sample company.

The reason why this paper considers adding *p* value is that the correlation between financial indicators is considered in the regression analysis of logical regression model, while the forward neural network is only the mapping from the input layer to the output layer through the middle layer and does not consider the correlation between financial indicators in the input layer. This may cause the overlapping information between the financial indicators of the input layer to affect the accuracy of the model, such as current ratio and quick ratio. Therefore, this paper uses the logistic regression model to modify the particle swarm neural network model, so as to make the model results more accurate.

The logistic regression model is used for modeling analysis below: let *p* be the probability of financial crisis, which is expressed by the following formula:

(8) $$\begin{array}{c} \text{Logit}\left(P\right)=\ln\left(\frac{P}{\left(1-P\right)}\right)=\alpha +\beta_{1}x_{1}+\beta_{2}x_{2}+\cdot \cdot \cdot +\beta_{n}x_{n}. \end{array}$$

Then, *P*=*e*^*α*+*β*_1_*x*_1_+*β*_2_*x*_2_+···+*β*_*n*_*x*_*n*_^/(1+*e*^*α*+*β*_1_*x*_1_+*β*_2_*x*_2_+···+*β*_*n*_*x*_*n*_^).

The *p* value represents the possibility. The greater the *p* value, the greater the possibility. If *p* is greater than a critical point, the event will basically occur. If *p* is less than the critical point, the possibility of event occurrence is relatively small. However, the definition of *p* value lacks theoretical basis and is highly subjective. As mentioned above, the logistic regression model is used for empirical analysis of 100 training samples, and the input data are 12 financial indicators. The obtained formula (9) is

(9) $$\begin{array}{c} P=\frac{e^{-1.582-1.279x_{1}+0.621x_{2}+\cdot \cdot \cdot -0.462x_{12}}}{\left(1+e^{-1.582-1.279x_{1}+0.621x_{2}+\cdot \cdot \cdot -0.462x_{12}}\right)}. \end{array}$$

The corresponding financial indicators of 100 training samples and 20 test samples are substituted to obtain the *p* value. According to the *p* value, it can be judged that the test sample has the possibility of financial crisis. When *p* is greater than a certain value, the company is more likely to fall into financial crisis, otherwise it means that the financial situation is good. The logistic regression model itself can be used as a financial early warning model, but the definition of *p* value is subjective, so the accuracy is not high. In this paper, the *p* value is used to modify the general particle swarm neural network model, so as to improve the accuracy of the model.

The general particle swarm optimization forward neural network model is used to empirically analyze the above samples. The sample data are 12 financial indicators. First, the neural network is initialized. There are 12 nodes in the input layer, 20 nodes in the middle layer, and 1 node in the output layer. If the output value is greater than 0.5, it means that the sample company is more likely to have a financial crisis, otherwise it means that there is less possibility of a financial crisis.

After initialization, the sample data are substituted into the model for empirical analysis in MATLAB.

As shown in Figure 7, it can be seen that with the increase of the number of iterations, the fitness of particles changes significantly, and the result is also decreasing. At the beginning of the iteration, the fitness is about 1.35, and when the number of iterations increases to 30, the fitness is reduced to about 0.7. When the number of iterations increases to 70, the fitness decreases to about 0.5 and remains stable.

From the output results in Figure 8, the model accuracy can reach 65%. This paper proposes two improved methods to improve the accuracy of the model.

1. Add the quantitative indicators of earnings management. At this time, the number of input layer nodes of the model is 13, including 12 traditional financial indicators and earnings management indicators, and the other parameters of the model remain unchanged.
2. The logistic regression model is used to modify the original model. The specific correction method is to substitute the sample data as above into the logistic regression model to obtain the *p* value and add the *p* value to the input layer of the neural network model. At this time, the number of input layer nodes of the model is 14, and the other parameters remain unchanged. Based on the above neural network model, the quantitative indicators of earnings management are added to the input layer, samples are empirically analyzed, and the results of the model are compared with the results of the above model.

In Figure 9, it can be found that, considering earnings management factors, the accuracy of the model is improved. In the model test samples without considering earnings management, the accuracy is 65% as shown in Figure 8. In the model test samples considering earnings management, the accuracy can reach about 70%.

On the basis of considering earnings management, the neural network model based on particle swarm optimization is modified by the logistic regression model, and the training samples and test samples are substituted into the modified model for empirical analysis. The results of modifying the model are shown in Figure 10.

It can be found that the alignment accuracy of the particle swarm neural network model modified by logistic regression model is significantly improved. In the model, the accuracy can reach 75%. The alignment accuracy of the modified particle swarm neural network model is obviously improved. It shows that, when using the particle swarm neural network to model and analyze the financial early warning of listed companies, adding earnings management indicators can improve the accuracy of particle swarm neural network model. In the demonstration, the correction of logistic regression model can also improve the accuracy of the particle swarm neural network financial early warning model. Compared with traditional methods, this paper adopts the particle swarm optimization algorithm. The system is initialized as a set of random solutions, and the optimal value is searched through iteration. Compared with the genetic algorithm, the particle swarm optimization algorithm is simple and easy to implement, and there is no need to adjust too many parameters. This greatly reduces the computational burden of the financial model and improves the accuracy of the early warning model.

## 5. Conclusion

The financial crisis of listed companies will cause great losses to stakeholders, so it is very important to establish a sound financial early warning mechanism. Based on the research of financial early warning models, this paper selects the particle swarm neural network model with the highest accuracy. In terms of data selection, in view of the widespread phenomenon of earnings management in listed companies, the earnings management indicators are substituted into the model. The empirical results show that the accuracy of the model considering earnings management factors is improved from 65% to 70%. In the process of modeling, this paper uses the logistic regression model to further modify the model. The empirical results show that the accuracy of the model can be improved from 70% to 75%. The final conclusion of this paper is that when using the particle swarm neural network to model and analyze the financial early warning of listed companies, adding earnings management indicators can improve the accuracy of particle swarm neural network model. In the demonstration, the use of logical regression model correction can also improve the accuracy of the particle swarm neural network financial early warning model. Compared with the traditional methods, the particle swarm optimization algorithm is used in this paper. The system is initialized as a set of random solutions, and the optimal value is searched through iteration. Compared with the genetic algorithm, PSO is simple and easy to implement, and there are not many parameters to be adjusted. This greatly reduces the computational burden of the financial model and improves the accuracy of the early warning model. However, the performance of particle swarm optimization algorithm used in this paper is not particularly good on some problems. The coding of parameter weight of early warning models needs to be further explored, and the selection of genetic operator is sometimes troublesome. Therefore, in the future research, we need to improve and supplement the data for the shortcomings of the algorithm.

## Figures and Tables

**Figure 1:** Forward neural network based on particle swarm optimization algorithm.

**Figure 2:** Interval span of each indicator.

**Figure 3:** Preprocessed data set.

**Figure 4:** F1-score curve of beta coefficient.

**Figure 5:** The proportion of the number of distance points in each interval and the cumulative proportion.

**Figure 6:** Test curve of transition probability parameters.

**Figure 7:** The fitness change curve during the operation of the particle swarm neural network model.

**Figure 8:** Output results of neural network model based on particle swarm optimization algorithm.

**Figure 9:** The output result of the model considering earnings management.

**Figure 10:** Output results of particle swarm optimization algorithm model modified by logistic regression model.

## Data Availability

The data used to support the findings of this study are available from the corresponding author upon request.
